# *Hypericum sampsonii* ameliorates radiodermatitis by inhibiting NLRP3 inflammasome activation

**DOI:** 10.1111/srt.70047

**Published:** 2024-09-23

**Authors:** Jiayu Liao, Zhihong Liu, Sumei Wu

**Affiliations:** ^1^ Department of Second Oncology Xinyu People's Hospital Xinyu China

**Keywords:** *Hypericum sampsonii*, NLRP3 inflammasome, radiation dermatitis, TLR4/NF‐κB

## Abstract

**Background:**

Radiodermatitis (RD) is an inflammatory lesion of skin mucosa caused by radiation, which causes itching and pain in patients' skin. *Hypericum sampsonii* has an anti‐inflammatory effect. This study aims to explore the potential effect and mechanism of *H. sampsonii* on RD.

**Materials and Methods:**

The RD model was established using X‐ray irradiation of mice and the pain response of mice under different treatment methods. Serum levels of IL‐1β, IL‐6, and TNF‐α were measured by ELSA. The RD cell model was constructed by RAW264.7 cell, *H. sampsonii* intervention was conducted, and the changes of the NLRP3 inflammasome in the cells were detected by qRT‐PCR. The cells were stimulated with LPS and the protein changes of TLR4/NF‐κB were investigated by Western Blotting.

**Results:**

*H. sampsonii* can better improve the skin status of RD mice, relieve pain, and reduce the secretion of serum inflammatory factors IL‐1β, IL‐6, and TNF‐α. *H. sampsonii* significantly down‐regulated the expression of NLRP3, Caspase‐1, pro IL‐1β, and IL‐1β. Lps‐induced activation of the TLR4/NF‐κB pathway promotes the expression of NLRP3 and pro‐IL‐1β, and *H. sampsonii* can inhibit this promotion.

**Conclusion:**

*H. sampsonii* may inhibit NLRP3 inflammatory vesicle activation via interfering with TLR4/NF‐κB signaling to reduce the inflammatory response in macrophages and thus play a role in the treatment of RD.

## 1 INTRODUCTION

Radiotherapy remains one of the most important treatments for malignant tumors, and it is estimated that up to 90% of patients treated with radiotherapy will develop varying degrees of erythema, desquamation, ulceration, and other radioactive skin lesions.^1^, ^2^ Radiodermatitis (RD) not only reduces the quality of life of patients, but also increases the painful experience of patients, and affects the treatment of patients in severe cases. The literature indicates that roughly half of all tumor patients undergoing radiotherapy develop grade III or non‐resolving RD, a condition that prompts the discontinuation of therapy and subsequently reduces survival duration. Presently, the most frequently employed clinical strategy for managing RD involves the application of topical medications.^3^, ^4^, ^5^ The relevant reports pointed out that Chinese medicinal materials have remarkable clinical efficacy in RD prevention and treatment.^6^, ^7^ It is of great clinical significance to explore effective Chinese medicinal materials for the prevention and treatment of RD, to clarify the etiology and pathogenesis, and to provide a theoretical basis and clinical basis for promoting the future treatment of RD.

*Hypericum sampsonii (* ***H. sampsomii***) is a perennial herb in the genus Hypericum Linn of the family Guttiferae, which is endemic to China. *H. sampsonii* is a traditional Chinese medicinal herb, which is included in the Compendium of Chinese Herbal Medicines and is used as a medicinal herb in folk medicine. According to the records of the Compendium of Materia Medica from the New, Hundred Herbs Mirror and Gleanings from the Compendium of Materia Medica, *H. sampsonii* has the effects of cooling the blood, stopping bleeding, clearing heat, and removing toxins, invigorating the blood and regulating menstruation, and dispelling wind and clearing the collaterals, and in recent years, it was found to have the effects of anti‐tumor, anti‐depressant, and antiviral, which has a wide prospect for development.^8^, ^9^ Studies have shown that *H. sampsonii* has important clinical value in anti‐tumor and anti‐inflammatory aspects. In the preliminary randomized herbal screening, our group found that the application of *H. sampsonii* impregnation solution to the radiotherapy area had a significant therapeutic effect on radiotherapy‐induced RD in tumor patients. However, the specific effect of *H. sampsonii* on RD and its mechanism are still unclear.

Studies have shown that the NOD‐like receptor family, pyrin domain‐containing protein 3 (NLRP3) inflammasome is closely related to the occurrence and development of many diseases.^10^, ^11^ NLRP3 inflammasome is a protein complex composed of the sensor NLRP3 pattern recognition receptor, apoptosis‐associated speck‐like protein containing a CARD domain (ASC), and the effector molecule pro Caspase‐1.^12^ Researchers have found that patients with Muckle‐Wells syndrome and familial Mediterranean fever and other genetic diseases have mutations in the NLRP3 gene on the chromosome, resulting in the NLRP3 inflammasome is always in an abnormally activated state, and many inflammatory factors, resulting in excessive inflammatory response.^13^, ^14^ Many studies have shown that traditional Chinese medicine can interfere with NLRP3, such as peony total flavonoids,^15^ naringin,^16^ and other Chinese herbal extracts can inhibit the activation of NLRP3 inflammasome axis and reduce NLRP3 expression.^17^ Therefore, it is tentatively speculated that *H. sampsonii* may be involved in the treatment of RD by modulating the activation of NLRP3 inflammasome.

This study aims to explore the effects of *H. sampsonii* on RD and NLRP3 inflammasome, providing new ideas for controlling the body's inflammatory response and clinical treatment.

## 2 MATERIALS AND METHODS

### 2.1 Study object

A total of 48 healthy adult male Sprague‐Dawley (SD) rats (Chengdu Yaokang Biotechnology Co., LTD.) with a body weight of 200–300 g and an age of 6–8 weeks were selected. They were fed regularly with a free diet and water. Adaptive feeding was performed for 2 weeks before the end of the experiment. This study was approved by Animal Ethics Committee of Xinyu People's Hospital.

### 2.2 Preparation of *H. sampsonii* immersion solution

The rhizomes of *H. sampsonii* were crushed using a crusher and poured into a large extraction tank, submerged in 95% ethanol solution, and soaked for 12 h. Then the temperature is set at 65°C, the first extraction is performed, the first impregnation is collected, and the 95% ethanol solution is poured into the remaining medicinal residue, followed by the second extraction. After reflux extraction for four times, the impregnation solution of each time was combined to obtain the total impregnation solution. Finally, *H. sampsonii* solution with a concentration of 1, 2, 4, 8, 16, 32 mg/mL wass prepared.

### 2.3 Grouping and intervention

All rats were divided into four groups with 12 rats in each group. One group was treated as healthy control group (HC) without treatment, and the other three groups were treated with X‐rays. Before irradiation, the mice were anesthetized, the hair on the left hind leg was uniformly plucked, and the markers were fixed with adhesive tape to ensure a uniform irradiated area. During irradiation, the rats were fixed, the right lower limbs were exposed, and other parts of the body were shielded with 6 MV X‐rays. After several pre‐experimental screenings, the irradiation program was determined: 2 m distance, 800 cGy/day for 5 days. The RD model mice were divided into a non‐interfering RD group, a *H. sampsonii* treatment group (HST), and a compound tea polyphenol ointment treatment group (CTP). The mice in the HST and CTP groups were uniformly coated with the drug with a sterile swab 1 day prior to irradiation, twice a day for 28 days. All mice were fed in the same way, and all skin conditions were observed at the end of the last dose of the drug and scored according to the scoring criteria for acute radiation response (RTOG/EORTC).^18^

### 2.4 Behavioral measurement of pain

The paw withdrawal mechanical threshold (PWMT) and paw withdrawal thermal latency (PWTL) of mice were measured sequentially at 1 d before modeling (0 d) and on days 1, 3, 7, 14, 21, and 28 after modeling, respectively, in strict accordance with the requirements of pain behavioral testing in animals.^19^ The experiment required the same tester to test uniformly at 4:00 pm every day, with a 1‐h interval between the two groups.

### 2.5 ELISA assay

On the morning of the 29th day, serum from the abdominal aorta of rats was collected, and after standing at room temperature for 60–120 min, supernatant was taken from 3500–4000 r/min and centrifuged for 10 min to extract the supernatant. The levels of IL‐1β, IL‐6, and TNF‐α in the supernatant were measured by Enzyme‐linked immunoassay (ELISA). The standards and samples to be tested were added into the blank control wells, standard wells, and samples to be tested wells, respectively, according to the instructions of ELISA kit (Invitrogen, USA). After the plate was heated and protected from light to develop the color, the reaction was terminated and the absorbance at 450 nm of each well was measured sequentially.

### 2.6 Cell culture and preconditioning

Mouse macrophage RAW264.7 was purchased from Wuhan University Cell Bank, China Typical Culture Collection Centre. The cells were firstly resuscitated, and the cell culture medium was replaced with DMEM complete culture medium (10% fetal bovine serum + 1% penicillin‐streptomycin‐neomycin), and then cultured in 37°C, 5% CO_2_ incubator, and the medium was changed every 2 days, and when 75%–80% fusion was reached, the cells were cultured in passaging culture, and the cells were ready for experiments at the age of 3–4 generations. Cells with good growth status were selected for RD modeling, and the cell culture medium was replaced with PBS solution and placed under a 2 cm thick liquid dressing. The distance from the radiation source to the cells was 100 cm, and the cells were irradiated according to the doses of 0.05, 0.1, 0.2, 0.4, and 0.8 Gy, respectively, and a total of 1 irradiation was performed at a dose rate of 300 MU/min. For lipopolysaccharide (LPS) treatment, LPS (1 μg/mL, Sigma, China) was added to all groups except the control group for 3 h of pretreatment, and then the LPS+HST group was incubated with corresponding drugs for 3 h.

### 2.7 CCK8 assay

After cell counting, the cells were inoculated into 96‐well plates, and after the cells were attached to the wall, the culture solution was aspirated, and different concentrations of *H. sampsonii* in the range of 1–32 mg/mL were added, and the solution was aspirated after incubation and observation for 24 h. Then the working solution was added into the corresponding wells according to the instructions of the CCK‐8 kit, and the absorbance at 450 nm was detected on an ELISA system. Then, according to the instructions of CCK‐8 kit, the equipped working solution was added to the corresponding wells, and the absorbance of each empty cell was detected on the enzyme‐linked immunoassay detector after 4 h to calculate the cell activity.

### 2.8 qRT‐PCR

In the morning of the 29th day, the skin tissues of rats were collected uniformly, and fasting was ensured for 12 h. Firstly, the rats were deeply anesthetized, and the skin tissues from the marked area of the right hind leg of the rats were taken, fixed with paraformaldehyde, and made into paraffin sections. To extract total RNA, the tissues were firstly milled and lysed to be added into EP tubes. Then lysis buffer was added according to the instructions of PureLink™ RNA Extract Kit (Thermo, USA), and the cells were completely lysed by repeated blowing with a pipette gun and transferred to a new EP tube. After centrifugation, 70% ethanol was added successively and Wash Buffe was used to purify RNA. Finally, the RNA was eluted with RNase‐Free Water and stored at −80°C for later use. For reverse transcription, the RNA samples to be measured were taken out, and the RNA with high purity was selected after detection and gDNA was removed. cDNA was obtained by reverse transcription according to the instructions of the Reverse Transcription Kit (Acres Biologicals, Hunan, China), and amplified according to the instructions of the PCR Kit (Next Sense Biotechnology Co., Ltd., Shanghai, China). Finally, the expression levels of the mRNAs were calculated using the 2^−ΔΔct^ method with GADPH as an internal reference.

### 2.9 Western Blotting

The tissue was split into cells, and the protein supernatant was extracted by adding RIPA lysate (BCA, Wuhan). The protein was transferred to the PVDF membrane by SDS‐PAGE electrophoresis and electro‐transfer device. PVDF membrane was soaked with 5% BSA, closed in a shaker at room temperature for 2 h, the primary antibody was added, incubated in a horizontal shaker at 4°C overnight, the secondary antibody was added and incubated at room temperature for 2 h, and the excess secondary antibody was washed away. Using β‐actin as the internal parameter, the gray value of the target strip was calculated.

### 2.10 Statistical analysis

Data were expressed as mean ± standard deviation (M ± SD), with statistical analysis conducted using SPSS17.0 software, and statistical charts generated using GraphPad Prism. The comparison among multiple sets of data was analyzed using One‐Way ANOVA. *p* < 0.05 was considered statistically significant.

## 3 RESULTS

### 3.1 Effect of *H. sampsonii* on radiation dermatitis

It was found that the dermatitis status of mice in the RD group was mostly at grade 4, in the DEX group it was mostly at grade 2–3, and inn the HST group it was mostly at grade 1 (Table 1). The PWTL and PWMT of mice in DEX group and HST group were significantly lower than those in RD group, and PWTL and PWMT had a significant improvement effect on the 8th day of treatment, and the effect of HST was slightly better than that of DEX (Figure 1A,B). Therefore, *H. sampsonii* has a good therapeutic effect on RD. In addition, further investigation revealed that the serum levels of IL‐1β, IL‐6, and TNF‐α were significantly increased in the mice after radiation exposure. Inflammatory factor levels were significantly reduced in both groups of rats after treatment, and the improvement in inflammatory factor levels was more pronounced in rats treated with *H. sampsonii* (Figure 1C–E).

**TABLE 1:** Grading of radiation dermatitis in mice of each group (sample, *n* = 12).

Group	Radiation dermatitis grades				
	Grade 0	Grade 1	Grade 2	Grade 3	Grade 4
HC	12	0	0	0	0
RD	0	0	1	3	8
RD+DEX	0	0	2	5	5
RD+HST	0	7	4	1	0

**FIGURE 1:** Effect of *H. sampsonii* on RD mice. *H. sampsonii* can reduce PMWT (A) and PTWL (B) in mice. *H. sampsonii* can reduce IL‐6 (C), IL‐1β (D), and TNF‐α (E) secretion in mouse serum.

### 3.2 Effect of *H. sampsonii* on cell activity

To further explore the effect of *H. sampsonii* on inflammatory factors, the RD cell model was constructed using macrophage RAW264.7, and the appropriate radiation dose was first screened. The selection of different radiation doses to irradiate cells showed that cell survival was severely affected by radiation doses higher than 200 cGY (Figure 2A). Therefore, screening irradiation doses in the range of 50–200 cGY for further study revealed that IL‐6 (Figure 2C) and TNF‐α (Figure 2D) concentrations were significantly increased (*p* < 0.05) at a radiation dose of 50 cGY, whereas there was no significant difference in IL‐1β concentration compared with the control group (*p* = 0.058, Figure 2B). Combining cell activity and the concentrations of inflammatory factor, the irradiation dose of 100 cGY was finally selected to construct the RD cell model. On this basis, exploring the effect of *H. sampsonii* on RAW264.7 cell activity revealed that the cell activity was significantly reduced when the concentration exceeded 4 mg/mL (*p* < 0.05, Figure 3A). In addition, it was found that when the concentration of *H. sampsonii* was 4 mg/mL, it significantly reduced the levels of IL‐1β, IL‐6, and TNF‐α in RD cells (*p* > 0.05, Figure 3B–D).

**FIGURE 2:** Establishment of macrophage RD model. Effects of different radiation doses on cell activity (A). Effects of different radiation metrology on IL‐1β (B), IL‐6 (C), and TNF‐α (D).

**FIGURE 3:** Toxic effects of Ingot on macrophages. Effect of *H. sampsonii* concentration on cell activity (A). Effect of *H. sampsonii* concentration on IL‐1β (B), IL‐6 (C), and TNF‐α (D).

### 3.3 Mechanism of action of *H. sampsonii*

Further exploration of the mechanism of action of *H. sampsonii* RD revealed that NLRP3 mRNA level was upregulated in skin tissues of RD mice (Figure 4A). Further analysis of the effect of *H. sampsonii* on NLRP3 inflammasome revealed that the relative expression of NLRP3 (Figure 4B), pro I IL‐1β (Figure 4C), Caspase‐1 (Figure 4E), and IL‐1β (Figure 4F) were all significantly reduced after the present *H. sampsonii* intervention, while the relative expression of pro Caspase‐1 relative expression was not significantly different (*p* = 0.171, Figure 4D). *H. sampsonii* is hypothesized to act by influencing the activation of the NLRP3 inflammasome. Based on the changes in NLRP3 inflammasome expression, it is hypothesized that *H. sampsonii* affects inflammasome activation through first signaling. Cells were stimulated using LPS to activate the NF‐κB signaling pathway. After the treatment of *H. sampsonii*, TLR4/NF‐κB protein levels in the skin tissue of RD mice were significantly reduced (Figure 5A,B). As shown in Figure 5C–F, LPS successfully induced the cells to activate TLR4, NF‐κB (p65), and upregulate the expression of NLRP3, pro IL‐1β, which was significantly suppressed after *H. sampsonii* intervention.

**FIGURE 4:** The impact of *H. sampsonii* on the NLRP3 inflammasome. *H. sampsonii* significantly reduced NLRP3 mRNA levels in mouse skin tissue (A) and macrophages (B). *H. sampsonii* significantly reduced pro IL‐1β (C), Caspase‐1 (E), and IL‐1β (F) mRNA levels in macrophages. *H. sampsonii* did not affect pro Caspase‐1 mRNA levels in macrophages (D).

**FIGURE 5:** Effect of *H. sampsonii* on TLR4/NF‐κB/NLRP3. *H. sampsonii* significantly reduced TLR4 (A) and p65 (B) protein levels in mouse skin tissue. *H. sampsonii* significantly inhibited LPS‐induced TLR4 (C) and p65 (D)activation. H. sampsonii reverses TLR4/NF‐κB‐promoted NLRP3 (E) and pro IL‐1β (F) upregulation.

## 4 DISCUSSION

According to the theory of Chinese medicine, RD belongs to hyperthermia and toxicity, so extracts or preparations of Chinese medicines with heat‐cleansing and detoxifying effects are mostly used, and the treatment of RD with Chinese medicines has achieved good therapeutic effects in clinical practice. In this study, the mouse RD model was first established, and it was observed that compared to compounded tea polyphenol ointment, *H. sampsonii* solution could better improve the skin condition and alleviate pain in RD mice. The levels of inflammatory factors IL‐1β, IL‐6, and TNF‐α were decreased after *H. sampsonii* intervention in RD mice. *H. sampsonii* has been reported to play an anti‐inflammatory role in LPS‐induced sepsis mice. Some studies have pointed out that the ingredient of *H. sampsonii* has anti‐inflammatory activity and great application potential in tumor‐related inflammation.^20^, ^21^ *H. sampsonii* has been reported to play an anti‐inflammatory role by inhibiting the secretion of inflammatory factors such as TNF‐α and IL‐6 in mice with LPS‐induced sepsis.^22^ The above suggests that *H. sampsonii* can inhibit the release of inflammatory factors and exert anti‐inflammatory effects to improve RD in mice, but the exact mechanism of the anti‐inflammatory effect of *H. sampsonii* is not clear.

In this study, it was also found that *H. sampsonii* significantly inhibited the secretion of macrophage inflammatory factors within a certain concentration range. Macrophages are the main inflammatory cells in skin injury, and activation of the NLRP3 inflammasome pathway of macrophages is a key pathway to activate the secretion of IL‐1β and other inflammatory factors. Several studies have reported that a variety of Chinese herbal medicines exert anti‐inflammatory effects by targeting NLRP3 inflammasome.^23^, ^24^ It has confirmed that the Chinese herb Xuan Lung Baidu significantly interferes with the NF‐κB and MAPK pathways, hinders the activation of NLRP3 inflammasome, and reduces the level of inflammatory factors.^25^ Xiang Lian Wan can inhibit the activation of NLRP3 inflammasome through TLR4/MyD88/NF‐κB signaling pathway and reduce the inflammatory response of ulcerative colon.^26^ Similarly, this study found that *H. sampsonii* significantly inhibited NLRP3 inflammasome activation and suppressed macrophage inflammatory factor secretion. Therefore, *H. sampsonii* is speculated to play an anti‐inflammatory role by influencing the activation of NLRP3 inflammasome in macrophages, inhibiting the release of inflammatory factors.

NLRP3 inflammasome activation requires two signaling stimuli, Signal 1 is the initiation of NLRP3 and pro‐IL‐1β transcription by the NF‐κB activation pathway and Signal 2 is the activation of inflammasome assembly.^27^ TLR4, p65 were found to be significantly inhibited by *H. sampsonii* in the RD mouse model. In addition, *H. sampsonii* did not affect pro Caspase‐1 mRNA levels. Therefore, it is speculated that *H. sampsonii* inhibits the activation of NLRP3 inflammasome through the first signals it acts on. To further confirm this conjecture, the present study used LPS to activate the NF‐κB signaling pathway and found that *H. sampsonii* significantly inhibited the activation of NF‐κB signaling and reduced NLRP3, pro IL‐1Βexpression. It has been suggested that caffeine inhibits the LPS‐induced macrophage MAPK/NF‐κB signaling pathway, suppresses the activation of the NLRP3 inflammasome, and improves bronchopulmonary dysplasia.^28^ Irisin has been found to ameliorate liver injury by inhibiting NF‐κB signaling, inhibiting the activation of NLRP3 inflammasome, and alleviating the release of LPS‐induced cellular inflammatory factors.^29^ Therefore, it is speculated that *H. sampsonii* is a pass interference TLR4/NF‐κB signal transduction that inhibits the activation of inflammasome and the release of inflammatory factors, thereby improving RD.

The above findings provide a potential mechanism for the treatment of RD by *H. sampsonii*, but only the NLRP3 inflammasome signaling pathway has been initially investigated, and the relevance of other inflammasomes, such as NLRP1, IPAF, and AIM2, has not been sufficiently studied. In addition, only the inflammatory factor IL‐1β was analyzed, and the other inflammatory factors activated by NLRP3 inflammasome and the deeper mechanisms of its influence have not been fully elucidated, therefore, more experimental studies are still needed to enrich and develop the theoretical basis for the treatment of RD in *H. sampsonii*, with a view to ultimately improving the prognosis of the disease.

## 5 CONCLUSION

In conclusion, the preliminary findings of this study suggest that *H. sampsonii* may inhibit the activation of NLRP3 inflammasome by interfering with the TLR4/NF‐κB signaling pathway, reduce the secretion of inflammatory factors from macrophages, and exert an anti‐inflammatory effect, thereby alleviating the skin condition and pain sensation of RD.

## CONFLICT OF INTEREST STATEMENT

The authors declare no conflicts of interest.

## ETHICS STATEMENT

This study was approved by Animal Ethics Committee of Xinyu People's Hospital.

## Data Availability

The data that support the findings of this study are available from the corresponding author upon reasonable request.
